# Clinical Outcomes and Predictors of Late Recurrence in Young Patients with Atrial Fibrillation after Catheter Ablation

**DOI:** 10.1155/2023/7892185

**Published:** 2023-05-29

**Authors:** Haonan Xu, Xiaowei Chen, Yubin Zhang, Kui Zhu, Jiangtao Zhao, Fen Qin, Hailong Tao

**Affiliations:** Department of Cardiology, The First Affiliated Hospital of Zhengzhou University, No. 1, Longhu Middle Ring Road, Zhengzhou 450000, China

## Abstract

**Background:**

Catheter ablation (CA) is an established treatment for atrial fibrillation (AF), but the recurrence of AF is not neglected. Young patients with AF were generally more symptomatic and intolerant to long-term drug treatment. We aim to explore clinical outcomes and predictors of late recurrence (LR) in AF patients younger than 45 years after CA to better manage them.

**Methods:**

We retrospectively studied 92 symptomatic AF patients who accepted CA from September 1, 2019, to August 31, 2021. Baseline clinical data (including N-terminal prohormone of brain natriuretic peptide, NT-proBNP), ablation outcomes, and follow-up outcomes were collected. Patients were followed up at 3, 6, 9, and 12 months. Follow-up data were available for 82/92 (89.1%) patients.

**Results:**

One-year arrhythmia-free survival was 81.7% (67/82) in our study group. Major complications occurred in 3/82 (3.7%) patients with an acceptable rate. The value of ln(NT-proBNP) (*P* = 0.025, odds ratio [OR] = 1.977, 95% confidence interval [CI] 1.087-3.596) and a family history of AF (*P* = 0.041, HR = 9.269, 95% CI 1.097-78.295) could independently predict AF recurrence. The ROC analysis of ln(NT-proBNP) showed that NT-proBNP greater than 200.05 pg/ml (area under the curve: 0.772, 95% CI 0.642-0.902, *P* = 0.001, sensitivity 0.800, specificity 0.701) was the cut-off point for predicting late recurrence.

**Conclusions:**

CA is a safe and effective treatment for AF patients younger than 45 years. Elevated NT-proBNP level and a family history of AF could be used as predictors for late recurrence in young patients. The result of this study may help us take more comprehensive management of those with high-recurrence risks to reduce disease burden and improve quality of life.

## 1. Introduction

Atrial fibrillation (AF) is one of the most prevalent cardiac arrhythmias in adults with a heavy health burden and is significantly influenced by age for prevalence and incidence [1]. Numerous studies of AF were focused on elderly patients, while the related observations in young patients are scarce [2–4]. An epidemiology study reported that the prevalence of AF was no more than 0.1% in patients younger than 45 years in the Chinese community population [5]. Young patients with AF were generally more symptomatic and intolerant to long-term drug treatment which was with higher adverse events when compared to catheter ablation [2].

Radiofrequency catheter ablation (RFCA) has been an established treatment for symptomatic and drug-refractory AF patients in the current guidelines [6, 7]. However, the recurrence after RFCA with AF is not neglected. The recurrence rate after RFCA varied from 20% to 45% among different studies [8–10]. Some risk factors associated with recurrent AF, such as type of AF, diabetes, and some echocardiographic parameters, are well established [8, 10, 11]. However, the research objects of present studies are mainly restricted to patients with an average age older than 60 years [12, 13]. The study focused on patients younger than 45 years is rare. Whether clinical outcomes and predictors of late recurrence in younger age patients with AF after RFCA differ from those in older age patients is unknown. A prognostic marker of young AF patients after ablation could help us take more comprehensive management of those with high-recurrence risks to reduce disease burden and improve quality of life. Based on the above considerations, our study was mainly designed to explore the clinical outcomes and predictors of late recurrence after RFCA in young patients with AF.

## 2. Materials and Methods

### 2.1. Study Population

We retrospectively collected 92 consecutive patients with AF younger than 45 years who accepted RFCA in our center from September 1, 2019, to August 31, 2021. Inclusion criteria were the symptomatic AF patients older than 18 years, those refractory to at least 2 antiarrhythmic drugs (AADs), and patients who accepted RFCA of AF for the first time. The exclusion criteria were the combination of left atrium (LA) thrombus, acute cardiac infarction, valvular atrial fibrillation, New York Heart Association (NYHA) III or IV class, and contradiction of anticoagulation. Finally, 2 patients were excluded for repeat ablation for AF and 4 were excluded for high NYHA class. The study was performed following the Declaration of Helsinki, and the study protocol was approved by the local ethics committee.

Demographic and clinical information at the hospital was collected including age, gender, type of AF, duration of AF, family history of AF, body mass index (BMI), alcohol consumption, smoking, and clinical comorbidities (diabetes, hypertension, thyroid disease, structural heart disease(SHD), and stroke). The definition of paroxysmal AF and persistent AF was referred to the 2020 ESC Guidelines for the diagnosis and management of atrial fibrillation [14]. Family history of AF was defined as at least one of the first-degree relatives (parents, siblings, children) having a medical history of AF. SHD was defined as the presence of hypertensive heart disease, coronary heart disease, cardiomyopathy, and grown-up congenital heart disease, as Hoffmann et al. previously described [15]. Laboratory and examination results were obtained such as the N-terminal prohormone of brain natriuretic peptide (NT-proBNP), left ventricular eject fraction (LVEF), and LA diameter. NT-proBNP was assayed in our center by commercially available assays in a blinded fashion. The blood samples were gathered in EDTA-anticoagulated tubes on admission. They were analyzed within 4 hours after collection. The HAS-BLED score and CHA_2_DS_2_-VASc score were computed for each patient.

### 2.2. Preprocedural Management

Transesophageal echocardiography and/or enhancement computer tomography was performed to exclude LA thrombus before RFCA. All AADs, except for amiodarone, were discontinued for at least 5 half-lives before ablation.

### 2.3. RFCA Procedure

All patients signed up for informed consent for RFCA procedures. Our standard ablation procedures were introduced in previous reports [16–18]. In brief, a decapolar catheter was placed in the coronary sinus through the left femoral vein. After the successful transseptal puncture through the right femoral vein, pulmonary venography was performed. Mapping and ablation were guided by the electroanatomical mapping system (CARTO, Biosense Webster, Diamond Bar, CA, USA). Circumferential pulmonary vein (PV) ablation was performed in all patients with limited radiofrequency energy of 35-40 W and a maximum ablation temperature of 45°C. The irrigation flow was 17 ml/min. The ablation procedure endpoint for paroxysmal AF was the isolation of all pulmonary veins. If typical atrial flutter was documented in the history or spontaneously occurred during the procedure, the cavotricuspid isthmus (CTI) was ablated. For patients with nonparoxysmal AF, additional linear ablation and/or superior vena cava (SVC) isolation was performed. The endpoint of linear ablation was the successful block of both sides. At the end of the RFCA, the PV isolation and bidirectional conduction block of each line would be evaluated.

### 2.4. Postablation Management

The first 3 months after the ablation procedure were named the blanking period. During this period, patients have been prescribed non-vitamin K antagonist oral anticoagulants (NOACs) and AADs. Amiodarone was given at the usual usage dose. If patients were contradicted with the amiodarone, propafenone was substituted. AADs were discontinued after 3 months postablation if there was no recurrence recorded.

### 2.5. Follow-Up

After discharge from the hospital, the patients were followed up every 3 months until 12 months. Major complications included hematoma, arteriovenous fistula, atrial-esophageal fistula, pulmonary vein stenosis, cardiac tamponade, etc. At each hospital visit, 24 h Holter recordings and ECG were performed. When patients experienced symptoms suggestive of AF recurrence, instruction was given to perform either ECG or 24 h Holter recording. Late recurrence was defined as any documented AF/atrial tachycardia (AT) episode >30 s after 3 months postablation. A repeat ablation procedure was recommended at least 3 months after the first time procedure when the restart of AADs or electrical cardioversion failed.

### 2.6. Statistical Analysis

Continuous variables are expressed as mean ± standard or median with 25th and 75th percentiles and compared using a *t*-test or rank-sum test. Categorical variables are expressed as frequencies (percentages) and compared using the chi-square test or Fisher's exact test. Kaplan-Meier curves were used to estimate 1-year arrhythmia-free survival. Predictors for the late recurrence of AF after RFCA were accessed by univariate and multivariate logistic regression models. Every parameter with a *P* value < 0.05 in the univariate analysis was considered for multivariate analysis. The value of NT-proBNP was transformed into a natural logarithm of NT-proBNP (ln(NT-proBNP)) to follow a normal distribution. For each selected variable, the odds ratio (OR) with 95% confidential interval (CI) and Wald test *P* value were displayed. The receiver operating characteristic (ROC) curves of significant variables in the multivariable model would be done to predict the relevant cut-off value. And the area under the curve (AUC) with a corresponding 95% CI and *P* value would be reported. The log-rank test was used to evaluate the difference in 1-year arrhythmia-free survival according to significant variables above or below the cut-off value. All data analyses were done using the IBM SPSS 26.0 software. A two-tailed *P* < 0.05 was considered statistically significant.

## 3. Results

After the 1-year follow-up, 4 patients did not finish the follow-up, and finally, 82 patients were analyzed. They were divided into the recurrent group and the nonrecurrent group.

### 3.1. Clinical Characteristics

The detailed baseline characteristics of patients in two study groups are presented in Table 1. Patients in the recurrent group had higher rates of SHD when compared to those in the nonrecurrent group (40.0% versus 11.9%, *P* = 0.026). A significantly higher rate of family history of AF was found in the recurrent group (26.7% versus 3%, *P* = 0.008). The NT-proBNP (878.7 ± 1131.5 pg/ml versus 244.7 ± 337.2 pg/ml, *P* < 0.001) was significantly higher in the recurrent group.

### 3.2. Procedure Results

Successful pulmonary vein isolation was achieved in all patients. CTI was performed in 12/15 (80.0%) patients in the recurrent group and 44/67 (65.7%) patients in the nonrecurrent group (*P* = 0.441). In patients with nonparoxysmal AF, additional linear and/or SVC isolation was performed in 7/8 (87.5%) patients in the recurrent group and 23/24 (95.8%) patients in the nonrecurrent group (*P* = 0.444) (Table 2).

### 3.3. Outcomes of Follow-Up

After 1-year follow-up, late recurrence was documented in 15/82 (18.3%) patients (Figure 1). Four patients in the recurrent group were readmitted. One of them accepted a repeat ablation, and the remaining three accepted electrical cardioversion. Three patients in the nonrecurrent group were readmitted for palpation, but no evidence of late recurrence was documented (Table 2).

### 3.4. Predictors of Late Recurrence of AF after RFCA

The detailed data is shown in Table 3. The univariate logistic regression model showed that the family history of AF (*P* = 0.008), SHD (*P* = 0.014), and ln(NT-proBNP) (*P* = 0.002) were statistically significant. The multivariate logistic regression model identified ln(NT-proBNP) (*P* = 0.025, OR =1.977, 95% CI 1.087-3.596) and a family history of AF (*P* = 0.041, OR =9.269, 95% CI 1.097-78.295) as predictors for late recurrence.

The ROC analysis of ln(NT-proBNP) showed that NT-proBNP greater than 200.05 pg/ml (sensitivity 0.800, specificity 0.701) was the cut-off point for predicting late recurrence (Figure 2). The AUC was 0.772 (95% CI 0.642-0.902, *P* = 0.001). Kaplan-Meier survival curves demonstrated that patients in the study group with NT-proBNP above the cut-off value had high-recurrence risks via the log-rank test (*P* < 0.001) (Figure 3).

### 3.5. Complications

Major complications occurred in 1/15 (6.7%) procedures in the recurrent group for hematoma. In the nonrecurrent group, major complications occurred in 2/67 (3.0%) procedures: 1 case of hematoma at the location of the femoral vein puncture and 1 case of arteriovenous fistula. No statistical difference was seen between the complications of the two groups (*P* = 0.459).

## 4. Discussion

This retrospective study discusses the clinical outcomes and predictors of late recurrence in young AF patients after RFCA. The main results of this study are shown as follows. First, RFCA is an effective and safe treatment choice for AF patients younger than 45 years, with satisfactory 1-year arrhythmia-free survival and an acceptable complication rate. Second, elevated NT-proBNP and a family history of AF could be used as predictors for late recurrence in young patients.

### 4.1. Clinical Outcomes of RFCA in Young Patients

Numerous random clinical trials and meta-analyses have investigated the initial choice of radiofrequency ablation or drug therapy for newly diagnosed atrial fibrillation with an average age above 60 years [2, 3]. Results of these studies showed that radiofrequency ablation is superior to antiarrhythmic drug therapy, for not only reducing all-cause rehospitalization but also improving the long-term quality of life for patients [19]. Our study focused on outcomes of RFCA in AF patients younger than 45 years. We found that 81.7% of patients maintained sinus rhythm after 1-year follow-up, and the complication rate is only 3.7%. Though the rehospitalization rate is high in recurrent patients (26.7%), the total rate of rehospitalization is low (8.5%). Similar results were found by Leong-sit et al. that after the follow-up of at least 28 months, patients younger than 45 years had a higher rate of arrhythmia-free survival without taking AADs (76%) compared to older patients, with a lower major complication rate (1.7%). Young patients with AF were generally more symptomatic and intolerant to long-term drug treatment. Therefore, RFCA is an effective and safe treatment choice for AF patients younger than 45 years, with satisfactory 1-year arrhythmia-free survival and an acceptable complication rate.

### 4.2. The Association of NT-proBNP and Late Recurrence of AF

Though RFCA now has become an effective and safe treatment selection for AF patients, the high-recurrence rate of AF after RFCA is a common medical conundrum [2, 20]. Several risk factors related to the recurrence of AF after RFCA have been identified in AF patients, such as type of AF, early recurrence of AF, and LA diameter [8, 17, 21]. However, predictors of late recurrence for young patients have been reported only in limited studies. Saguner et al. reported that obesity (BMI > 30 kg/m^2^) and structural heart disease independently predicted AF recurrence in young patients [22]. Moran et al. found that the only predictor of AF recurrence was hypertrophic cardiomyopathy in patients under 40 years old [23].

In our study, elevated NT-proBNP could independently predict late recurrence, with a cut-off value of 200.05 pg/ml. NT-proBNP is mainly secreted by cardiomyocytes of the left ventricle (LV), which is increased with age [24–26]. NT-proBNP is an indicator of heart failure, and it is also currently used at high rates in patients with new-onset and recurrent AF even without underlying heart disease [27, 28]. Pressure or volume overload and myocardial stretch could stimulate the secretion of NT-proBNP [24]. It is reported that NT-proBNP could also be produced by the atrial wall in a recent study [29]. Structural and electrical LA remodeling caused by irregular atrial contraction and increased atrial stretch of AF could stimulate the secretion of NT-proBNP [30, 31]. The increased filling pressure of both LA and LV resulting from cardiac dysfunction and hypertension could also increase the secretion of NT-proBNP [31]. NT-proBNP has been studied to be a risk factor for AF recurrence after RFCA and electrical cardioversion in several studies [21, 32]. Our study showed the same finding that the increased NT-proBNP level was the predictor of AF recurrence after RFCA in young patients which indicated that heavy atrial remodeling and overload volume and pressure were common in young patients with AF recurrence.

Based on the above discoveries, early treatment to decrease the secretion of NT-proBNP may be beneficial to prevent AF recurrence in young patients. Recent studies found that the combination of irbesartan or losartan with low-dose amiodarone could help to maintain sinus rhythm by inhibiting left atrial enlargement and decreasing atrial stretch and filling pressure which decreases the production of NT-proBNP [33, 34]. Results of the ARREST-AF study proved that better management of risk factors like hypertension, diabetes, and obesity was linked with a lower AF recurrence rate after catheter ablation by decreasing LA remodeling [35]. Less remodeling could reduce myocardial stretch and the secretion of NT-proBNP of LA. However, further clinical studies are needed.

Though several studies have identified that elevated baseline NT-proBNP is a predictor for AF recurrence after RFCA, same as the finding in this study, no agreement has been reached as to the predictive value of baseline NT-proBNP [21, 24]. The study of Giannopoulos et al. found no significant association between AF recurrence and NT-proBNP after adjusting for variables [36]. Ma et al. found that NT-proBNP was linked with AF recurrence in patients with persistent AF after RFCA but not found in patients with paroxysmal AF [37]. Shunsuke et al. found that BNP was a more helpful indicator of AF recurrence for patients with baseline rhythm of AF. The aim of our study focused on predictors irrespective of AF type, and there was no difference in AF type between the two groups in our study. The time of collecting blood samples and assaying for NT-proBNP is also controversial. Most studies focused on baseline NT-proBNP before RFCA like our study [24]. Others like Elmas et al. found that NT-proBNP was the predictor of AF recurrence when blood samples were obtained the day after ablation but not preablation [38].

### 4.3. The Association between Family History and Late Recurrence of AF

The study of Gourraud et al. found that a family history of AF was more commonly seen in young patients [39]. Kapur et al. also demonstrated that a positive family history of AF was related to a higher arrhythmia recurrence rate in patients with persistent AF (*P* = 0.04) [40]. In this study, we found similar results in that young patients who had a family history of AF had a higher recurrence risk after RFCA. Furthermore, a family history of AF may reflect a genetic disease in young patients, such as Brugada syndrome and long QT syndrome, because the major cause of AF in the young population are cardiomyopathy, ion-channel disease, and genetic factors [39, 41, 42]. Shoemaker et al. found an increased risk of recurrence after RFCA of AF when AF susceptibility alleles at the 4q25/PITX2 locus were identified [43]. A genetically different phenotype may be associated with arrhythmia recurrence, but there remained a lot that was still unclear and needed to be defined. Genetic testing may contribute to discovering these genetic variants, but it may be hard to commonly utilize them in clinical practice.

### 4.4. Clinical Implication

This study demonstrated that RFCA is a safe and effective treatment choice for AF patients younger than 45 years, with a satisfactory 1-year arrhythmia-free survival and acceptable complication rate. Elevated NT-proBNP level and a family history of AF were associated with higher recurrence risks for patients younger than 45 years. The results of our study may help us to inform these young patients about the risk-benefit ratio of the RFCA to help them choose treatment strategies in the future.

### 4.5. Limitations

First, this study is a retrospective and single-center study with a small-size population and a limited ability to form a conclusion. Second, some recurrences of spontaneous arrhythmia without obvious symptoms are hard to detect by our present follow-up designs. This may underestimate the recurrence rate of AF. A prospective, large enrollment study with a more sensitive design of follow-up is needed to further explore this issue. Finally, some parameters related with AF recurrence were not measured in this study, such as early recurrence and uric acid/albumin ratio. We could not find whether these risk factors were still associated with AF recurrence in young patients [44, 45].

## 5. Conclusions

RFCA is a safe and effective treatment for AF patients younger than 45 years. Elevated NT-proBNP level and a family history of AF could be used as predictors for late recurrence in young patients.

## Figures and Tables

**Figure 1:** Kaplan-Meier survival curves of arrhythmia-free survival in young patients.

**Figure 2:** (a) The receiver operating characteristic (ROC) curves of NT-proBNP in patients ≤ 45 years. The cut-off value is 200.05 pg/ml (sensitivity 0.800, specificity 0.701). (b) The distribution of the NT-proBNP values in the two groups according to the cut-off value. NT-proBNP: N-terminal prohormone of brain natriuretic peptide; AUC: area under the curve; CI: confidence interval.

**Figure 3:** The Kaplan-Meier survival curves of arrhythmia-free survival by the cut-off value of the N-terminal prohormone of brain natriuretic peptide in patients ≤ 45 years.

**Table 1:** Baseline clinical characteristics of the study groups.

Characteristic	All (*n* = 82)	Recurrent (*n* = 15)	Nonrecurrent (*n* = 67)	*P* value
Age (years)	38.0 ± 6.3	38.3 ± 6.0	37.9 ± 6.4	*P* = 0.923
Gender				
Male	63 (76.8%)	9 (60.0%)	54 (80.6%)	*P* = 0.171
Female	19 (23.2%)	6 (40.0%)	13 (19.4%)	
AF				
Paroxysmal AF	50 (61.0%)	7 (46.7%)	43 (64.2%)	*P* = 0.209
Nonparoxysmal AF	32 (39.0%)	8 (53.3%)	24 (35.8%)	
Duration (months)	22.9 ± 36.6	17.2 ± 19.2	24.2 ± 39.5	*P* = 0.809
Family history	6 (7.3%)	4 (26.7%)	2 (3.0%)	*P* = 0.008
BMI (kg/m^2^)	25.5 ± 3.5	24.2 ± 3.5	25.7 ± 3.4	*P* = 0.109
Smoking	16 (19.5%)	1 (6.7%)	15 (22.4%)	*P* = 0.304
Alcohol consumption	10 (12.2%)	1 (6.7%)	9 (13.4%)	*P* = 0.774
Comorbidities	35 (42.7%)	9 (60.0%)	26 (38.8%)	*P* = 0.134
Hypertension	11 (13.4%)	0 (0%)	11 (16.4%)	*P* = 0.205
Diabetes	6 (7.3%)	1 (6.7%)	5 (7.5%)	*P* = 1.000
OSAHS	9 (11.0%)	1 (6.7%)	8 (11.9%)	*P* = 0.894
Thyroid disease	5 (6.1%)	2 (13.3%)	3 (4.5%)	*P* = 0.225
Stroke	3 (3.7%)	0	3 (4.5%)	*P* = 1.000
SHD	14 (17.1%)	6 (40.0%)	8 (11.9%)	*P* = 0.026
LA diameter (mm)	37.1 ± 7.5	38.6 ± 7.2	36.8 ± 7.6	*P* = 0.324
LVEF (%)	61.6 ± 5.5	60.6 ± 7.7	61.9 ± 5.0	*P* = 0.759
NOACs	80 (97.6%)	15 (100%)	65 (97.0%)	*P* = 1.000
AAD	79 (96.3%)	13 (86.7%)	66 (98.5%)	*P* = 0.085
Class I AAD	2 (2.4%)	1 (6.7%)	1 (1.5%)	
Class II AAD	1 (1.2%)	0	1 (1.5%)	
Class III AAD	76 (92.7%)	12 (80%)	64 (95.5%)	
Class IV AAD	0	0	0	
CHA_2_DS_2_-VASc score	1 (0, 1)	1 (0, 1)	1 (0, 1)	*P* = 0.607
HAS-BLED score	0 (0, 1)	0 (0, 0)	0 (0, 1)	*P* = 0.063
NT-proBNP (pg/ml)	360.7 ± 612.2	878.7 ± 1131.5	244.7 ± 337.2	*P* = 0.001

Values are means ± standard deviations or medians with 25th and 75th percentiles and frequencies (percentages). AF: atrial fibrillation; BMI: body mass index; OSAHS: obstructive sleep apnea-hypopnea syndrome; SHD: structural heart disease; LA: left atrium; LVEF: left ventricular eject fraction; NOACs: non-vitamin K antagonist oral anticoagulants; AADs: antiarrhythmic drugs.

**Table 2:** Procedure outcomes.

	Recurrent (*n* = 15)	Nonrecurrent (*n* = 67)	*P*
PVI attempted	15/15 (100%)	67/67 (100%)	*P* = 1.000
Ablation of CTI	12/15 (80.0%)	44/67 (65.7%)	*P* = 0.441
Additional ablation	7/8.(87.5%)	23/24 (95.8%)	*P* = 0.444
Complications	1/15 (6.7%)	2/67 (3.0%)	*P* = 0.459
Rehospitalization	4/15 (26.7%)	3/67 (4.5%)	*P* = 0.023

Additional ablation: additional linear and/or SVC isolation for nonparoxysmal AF patients; PVI: pulmonary vein isolation; CTI: cavotricuspid isthmus.

**Table 3:** Univariate and multivariate logistic regression analyses of the recurrence of AF in young patients.

	Univariate OR	*P*	Multivariate OR	*P*
Male	2.769 (0.836-9.170)	0.095		
AF duration (months)	0.993 (0.973-1.014)	0.506		
Nonparoxysmal AF	2.048 (0.661-6.343)	0.214		
Family history	11.818 (1.927-72.480)	0.008	9.269 (1.097-78.295)	0.041
BMI (kg/m^2^)	0.865 (0.719-1.042)	0.127		
OSAHS	0.527 (0.061-4.563)	0.561		
SHD	4.917 (1.381-17.504)	0.014	2.411 (0.520-11.172)	0.261
LVEF (%)	0.962 (0.877-1.056)	0.419		
LA diameter (mm)	1.030 (0.961-1.104)	0.398		
ln(NT-proBNP)	2.401 (1.396-4.128)	0.002	1.977 (1.087-3.596)	0.025

AF: atrial fibrillation; OR: odds ratio; BMI: body mass index; OSAHS: obstructive sleep apnea-hypopnea syndrome; SHD: structural heart disease; LVEF: left ventricle eject fraction; LA: left atrium.

## Data Availability

The data presented in this study are available on reasonable request from the corresponding author.
